# Tetrandrine Suppresses Lipopolysaccharide-Induced Microglial Activation by Inhibiting NF-κB and ERK Signaling Pathways in BV2 Cells

**DOI:** 10.1371/journal.pone.0102522

**Published:** 2014-08-12

**Authors:** Yalong Dang, Yongsheng Xu, Wentao Wu, Weiyi Li, Yanran Sun, Jing Yang, Yu Zhu, Chun Zhang

**Affiliations:** 1 Department of Ophthalmology, the First Affiliated Hospital of Zhengzhou University, Zhengzhou City, Henan Province, People's Republic of China; 2 Clinical Stem Cell Research Center, Peking University Third Hospital, Beijing, People's Republic of China; 3 Department of Ophthalmology, Peking University Third Hospital, Beijing, People's Republic of China; Robert Debre Hospital, France

## Abstract

**Background and Objective:**

Tetrandrine (TET) is a bisbenzylisoquinoline alkaloid extracted from *Stephania tetrandra* Moore. Recent studies have suggested that TET can reduce the inflammatory response in microglia, but the mechanisms remain unclear. The aim of this study is to investigate whether TET can inhibit lipopolysaccharide (LPS)-induced microglial activation and clarify its possible mechanisms.

**Study Design/Materials and Methods:**

Cell viability assays and cell apoptosis assays were used to determine the working concentrations of TET. Then, BV2 cells were seeded and pretreated with TET for 2 h. LPS was then added and incubated for an additional 24 hours. qRT-PCR and ELISA were used to measure the mRNA or protein levels of IL1*β* and TNFα. Western blotting was utilized to quantify the expression of CD11b and cell signaling proteins.

**Results:**

TET at optimal concentrations (0.1 µM, 0.5 µM or 1 µM) did not affect the cell viability. After TET pretreatment, the levels of IL1*β* and TNFα (both in transcription and translation) were significantly inhibited in a dose-dependent manner. Further studies indicated that phospho-p65, phospho-IKK, and phospho-ERK 1/2 expression were also suppressed by TET.

**Conclusions:**

Our results indicate that TET can effectively suppress microglial activation and inhibit the production of IL1*β* and TNFα by regulating the NF-kB and ERK signaling pathways. Together with our previous studies, we suggest that TET would be a promising candidate to effectively suppress overactivated microglia and alleviate neurodegeneration in glaucoma.

## Introduction

Microglia constitute a unique population of immune cells in the CNS. They are distributed throughout the brain and retina, represent approximately 12% of the adult brain cells, and play a pivotal role in the innate immune response [1]. In normal conditions, microglia support synaptogenesis through the local synthesis of neurotrophic factors [2], [3] and the regulation of synaptic transmission and remodeling [4],[5]. In response to acute neurodegenerative disease, they transform from a ramified basal homeostatic phenotype to an activated phagocytic phenotype and release pro-inflammatory mediators, such as IL1β and TNFα. This acute neuroinflammatory response is generally beneficial to the CNS because it tends to minimize further injury and contributes to the repair of damaged tissues [6], [7], [8], [9]. In contrast, chronic neurodegenerative diseases, including Alzheimer's disease (AD), multiple sclerosis (MS), Parkinson's disease (PD), amyotrophic lateral sclerosis (ALS), and glaucoma are recognized to be associated with chronic neuroinflammation. Long-term activation of microglia is the most prominent feature of chronic neuroinflammation. Sustained release of inflammatory mediators by activated microglia may induce increased oxidative and nitrosative stress, always leading to neurotoxic consequences [10].

Glaucoma is a chronic neurodegenerative disease [11]. The progressive degeneration of retinal ganglion cells (RGCs) and sustained loss of the visual field are its remarkable characteristics [12]. Recent studies suggested that activated microglia participate in the pathological course of glaucomatous optic injury with adverse consequences [13], [14], and reduced microglial activation was associated with alleviating optic nerve and retinal neurodegeneration [15].

Tetrandrine(TET) [16], a bisbenzylisoquinoline alkaloid extracted from *Stephania tetrandra* Moore, has a variety of biologic activities and has been used to treat patients with tumors [17], hypertension [18], fungal infection [19] and silicosis [20] for decades. Recently, in vitro and in vivo studies have suggested that TET reduced the inflammatory response in macrophages by inhibiting the production of chemokines and cytokines [21]. Other studies also reported that TET decreased the production of TNFα, IL1β, IL6 and NO in activated microglia by inhibiting the NF-κB signaling pathway [22], [23].

Mitogen-activated protein kinases (MAPKs), including ERK 1/2, JNK, and p38, are a group of signaling molecules, and play an important role in pro-inflammatory cytokine expression [24]. Previous studies demonstrated that the up-regulation of the MAPK signaling pathway was involved in various models of microglial activation [25], [26]. Further studies also suggested that the effective inhibition of the MAPK pathway could decrease the production of pro-inflammatory cytokines and thus be beneficial for neuronal survival [27]. However, it is unclear whether TET could affect the MAPK signaling pathway in activated microglia. In this study, we investigated the inhibitory function of TET in LPS-activated microglia and clarified its possible mechanisms.

## Methods

### 2.1 Experimental procedures

Tetrandrine (Sigma, European Pharmacopoeia (EP) Reference Standard, purity>99%) was dissolved in 0.1N HCl and adjusted to pH 7.3. Then, it was diluted to give a 1 mM concentrated stock solution in sterile PBS and filtrated with a nitrocellulose filter with a pore size of 0.22 µm (Millipore). When in use, the stock solution was further diluted to the desired concentrations with culture medium. Cell viability assays and cell apoptosis assays were used to identify the working concentrations of TET. BV2 cells were seeded, pretreated with TET at variable concentrations for 2 hours, and LPS (Sigma, final concentration: 1 µg/ml) was then added to the medium. The plates were incubated for an additional 24 hours (Total 26 hours) in the presence of TET and 10% FBS. Finally, the supernatant and cells were harvested for further analysis. qRT-PCR and ELISA were used to measure the expression of IL1*β* and TNFα. Western blotting was utilized to detect the expression of CD11b and cell signaling proteins.

### 2.2 Cell Culture

Immortalized mouse BV2 microglial cell lines were purchased from the Cell Resource Center, Institute of Basic Medical Science, Peking Union Medical University (Beijing, China). Cells were maintained in Dulbecco's Modified Eagle's Medium(High Glucose, Gibco) with 10% heat-inactivated fetal bovine serum (FBS, Gibco) at 37°C in a humidified incubator under a 95%/5% (v/v) mixture of air and CO_2_. When cells were grown to approximately 80% confluence, they were digested with trypsin (Gibco) and passaged for additional experiments.

### 2.3 Cell Viability Assay

Cell viability was evaluated by the Cell Counting Kit (Dojindo Laboratories). Briefly, 100 µl of cell suspension (5×10^4^ cells/ml) was seeded into 96-well plates overnight. TET was added at various concentrations for 2 hours (0 µM, 0.1 µM, 0.5 µM, 1 µM, 2 µM, 5 µM, and 10 µM). Then, LPS (final concentration: 1 µg/ml) was added to each well and incubated at 37°C for 24 hours (total 26 hours) in the presence of TET and 10% FBS. Thereafter, 10 µl of CCK-8 solution was added to each well and incubated for an additional 2 hours. Absorbance was measured at 490 nm using a microplate reader (Sunrise, Tecan). Optical density was identified as the relative numbers of viable cells. All the experiments were performed in triplicate.

### 2.4 Cell Apoptosis Assay

To investigate whether TET has cytotoxicity, cells were measured by a fluorescence activated cell sorter (FACS, BD Bioscience) using an Annexin V-FITC Apoptosis Kit (Dojindo Laboratories) according to the manufacturer's protocol.

Briefly, 10^6^ BV2 cells were seeded into 60 mm TC-treated dishes overnight, then pretreated with various concentrations of TET (0.1 µM, 0.5 µM, 1 µM, 2 µM, 5 µM, and 10 µM) for 2 hours. LPS (final concentration: 1 µg/ml) was added to each plate and incubated at 37°C for 24 hours (total 26 hours) in the presence of TET and 10% FBS. Cells were digested, resuspended in Annexin V binding buffer (adjusted cell density to 10^6^/ml). Approximately 200 µl of cell suspension was aspirated to a new tube. Then, 5 µl of AnnexinV-FITC solution was added. After incubating for 15 min at room temperature, 5 µl of propidium iodide (PI) was also added. Finally, cells were analyzed by FACS. An unstained cell suspension was prepared in PBS, which acted as a negative control for FACS. All tests were conducted in triplicate.

### 2.5 Enzyme-linked Immunosorbent Assay, ELISA

Protein levels of IL1*β* and TNFα in supernatant were measured by an ELISA kit (BD Bioscience) according to the manufacturer's protocol. Briefly, 3×10^6^ cells were seeded into 100 mm TC-treated dishes overnight and then pretreated with TET at different working concentrations (0.1 µM, 0.5 µM, 1 µM) for 2 hours. After that, the cells were stimulated with LPS (final concentration: 1 µg/ml) for 24 hours in the presence of TET and 10% FBS. Finally, the supernatant was collected and stored at −80°C, the cells were lysed for RNA extraction and Western blotting. All tests were performed in triplicate.

### 2.6 Reverse Transcriptase-Polymerase Chain Reaction (RT-PCR)

Total RNA was extracted with TRIzol Reagent (Invitrogen). Reverse-transcriptase and quantitative PCR were performed on the SuperScript One-Step RT-PCR System (Applied Biosystems), according to the manufacturer's instructions. One microgram of RNA template was reverse-transcribed using a PrimeScript RT Master Mix Kit (TaKaRa Bio Inc, Dalian, China) according to the manufacturer's protocol. Subsequently, 2 µl of cDNA solution of each sample were subjected to real-time polymerase chain reaction in a 20-µL reaction mixture containing 10 µl of 2× SYBR Premix Ex Taq II, 0.4 µl of 50× ROX Reference Dye, 0.8 µl of PCR Forward Primer (Final concentration: 0.4 µM), 0.8 µl of PCR Reverse Primer (Final concentration: 0.4 µM), and 6 µl of dH_2_O. Triplicate PCR reactions were prepared for each cDNA sample. β-actin was used as an internal standard. Blank controls (PBS instead of cDNA template) were performed in each run. Amplification was not found in the blank controls. The primers designed for quantitative PCR are listed in Table 1.

**Table 1:** Primers Used for Quantitative RT-PCR.

Gene	Forward Primer 5′-3′	Reverse Primer 5′-3′	Accession	Size (bp)
**IL1β**	AATGACCTGTTCTTTGAAGTTGA	TGATGTGCTGCTGCGAGATTTGAAG	NM_008361.3	115
**TNFα**	GAAAAGCAAGCAGCCAACCA	CGGATCATGCTTTCTGTGCTC	NM_001278601.1	106
**β-actin**	TCCTCCTGAGCGCAAGTACTCT	GCTCAGTAACAGTCCGCCTAGAA	NM_007393.3	153

### 2.7 Western blot analyses

Cells were harvested and homogenized in ice-cold Cell Extraction Buffer (Bioworld) supplemented with 1 mM phenylmethanesulfonyl fluoride (PMSF, Sigma). Upon centrifugation at 12000 g for 15 min at 4°C, the supernatant was collected and protein concentration was quantified by a Bicinchoninic Acid Protein Assay Kit (Bioworld) according to the manufacturer's instructions. Approximately 30 µg of proteins from each sample were loaded into the wells of a 10% SDS-PAGE gel for electrophoresis followed by electro-transfer to polyvinylidene difluoride membranes (GE). The membranes were blocked by StartingBlock T20 (Pierce Biotechnology) prior to incubation in primary antibodies: CD11b (1∶300, #ab8878, AbCam), p-P65 (1∶1000, #13346, Cell Signaling), P65 (1∶800, #ab7970, AbCam), p-IKK (1∶1000, #2697, Cell Signaling), IKK(1∶250, #ab54626, AbCam), p-ERK (1∶2000, #4370, Cell Signaling), ERK(1∶1000, #4696,Cell Signaling), p-JNK (1∶1000, #9251, Cell Signaling), JNK(1∶1000, #9252, Cell Signaling), p-P38 (1∶1000, #4511, Cell Signaling), and P38(1∶500, #9212, Cell Signaling) and β-actin (1∶400, #ab3280, AbCam) overnight at 4°C. After thorough washing, the membrane was incubated with horseradish peroxidase (HRP) conjugated secondary antibody (1∶1000, A0208, Beyotime, Haimen, China) and developed with Supersignal West Dura Extended Duration Substrate (Thermo Scientific Pierce) and imaged using an Autochemie System (UVP, Upland, CA). The relative integrated intensity for CD11b, p-P65, P65, p-IKK, IKK, p-ERK, ERK, p-JNK, JNK, p-P38, and P38 was normalized to that of β-actin in the same sample. All tests were conducted in triplicate.

### 2.8 Statistical analyses

Results were expressed as the mean ±S.D. from three independent experiments. The statistical significance of the differences was established by one-way analysis of variance followed by Dunnett's test. Two-tailed values of *P*<0.05 were considered to be statistically significant.

## Results

### 3.1TET has no cytotoxicity at optimal concentrations

#### 3.1.1 TET with optimal concentrations did not influence cell viability

Cells were pretreated with TET (0.1 µM to 10 µM) for 2 hours followed by LPS (1 µg/ml) application for another 24 hours. As shown in Fig. 1, we found that TET has no cytotoxicity in the concentration range from 0.1 µM to 1 µM.

**Figure 1:** Effect of TET on the cell viability of BV2 cells. BV2 cells were treated with TET at various concentrations for 2 h. Then, LPS was added to each well and incubated at 37°C for an additional 24 h. Cell viability was measured by CCK-8 assay. Results were expressed as a percentage of the control cultures and the mean ±S.D. from three independent experiments performed in triplicate. * *P*<0.05 compared with the LPS (−) TET (−) group.

#### 3.1.2 TET with optimal concentrations did not increase the percentage of cell apoptosis

As shown in Fig. 2, after 2 hours of TET pretreatment and 24 hours of LPS stimulation, TET at 0 µM (LPS−), 0 µM, 0.1 µM, 0.5 µM, 1.0 µM, 2.0 µM, 5.0 µM, and 10.0 µM resulted in (10.7±2.6)%, (8.9±1.9)%, (11.9±2.3)%, (12.7±3.1)%, (13.4±2.8)%, (27.4±5.2)%, (96.8±1.17)% and (97.7±3.42)% of apoptotic cells (mean±S.D), respectively. As shown in Fig. 2e, statistical analysis revealed TET with optimal concentrations (0.1 µM, 0.5 µM, 1.0 µM) did not induce cell apoptosis. These results were consistent with the CCK-8 assay. Therefore, TET in a concentration range of 0.1 µM, 0.5 µM and 1 µM was used in the subsequent studies.

**Figure 2:** The percentage of apoptotic BV2 cells induced by TET. BV2 cells were treated with TET at various concentrations for 2 h; then, LPS was added to each plate and incubated at 37°C for an additional 24 h. Fig. 2a–2f: Cell apoptosis was monitored by FACS using an Annexin V-FITC Apoptosis Kit. Fig. 2e: Results were expressed as a percentage of apoptosis cells and were the mean ± S.D. from three independent experiments performed in triplicate. * *P*<0.05 compared with the LPS(−)TET(−) group.

### 3.2 TET inhibited LPS-induced microglial activation

BV2 cells were pretreated with TET (Final concentration: 0.1 µM, 0.5 µM and 1 µM) for 2 hours before the application of LPS (1 µg/ml). A total of 26 hours later, the cells were imaged under a phase-contrast microscope (Olympus) and then lysed for the extraction of total proteins and the detection of CD11b expression.

#### 3.2.1 Morphological Changes

Generally, the basal homeostatic microglia have a ramified shape. Once activated, the cells quickly convert to round or amoeboid shapes within two hours [28]. In this study, as shown in Fig. 3, approximately (75.2±6.2)% of BV2 cells (mean±S.D) displayed round or amoeboid shapes in the control group. After LPS stimulation, (94.5±2.6)% of BV2 cells (mean±S.D) were activated in the LPS group. In contrast, at the end of this experiment, (89.4±4.6)%, (86.2±2.9)%, and (80.7±3.9)% of BV2 cells (mean±S.D) showed round or amoeboid shapes in the 0.1 µM, 0.5 µM, and 1 µM TET groups, respectively (*P* = 0.781, *P* = 0.045, *P* = 0.033, respectively). (Figure 3)

**Figure 3:** Morphological changes of BV2 cells with or without TET pretreatment (scale bar: 300 µm). BV2 cells were treated with TET at working concentrations for 2 h. Then, LPS was added to each plate and incubated at 37°C for an additional 24 h. Fig. 3a shows the morphological changes of BV2 cells with or without TET pretreatment. Red arrows indicate the activated BV2 cells. Black arrows indicate the basal homeostatic BV2 cells. Fig. 3b: Activated cells and total cells were counted under a phase contrast microscope. Results were expressed as the percentage of activated cells and were the mean ± S.D. from three independent experiments performed in triplicate. * *P*<0.05 compared with the LPS(+)TET(−) group.

#### 3.2.2 CD11b expression

CD11b, a molecular marker of microglia, is expressed in both activated and basal homeostatic microglia. A recent study indicated that CD11b would be up-regulated in activated microglia when compared with basal homeostatic cells [29]. In our study, we considered the expression of CD11b to be an indicator of microglial activation. As shown in Fig. 4, 1 µg/ml of LPS significantly stimulated the CD11b expression of BV2 cells, but pretreatment with TET inhibited these effects in a dose-dependent manner.

**Figure 4:** Effect of TET on CD 11b expression in BV2 cells. BV2 cells were treated with TET at working concentrations for 2 h. Then, LPS was added to each plate and incubated at 37°C for an additional 24 h.The cells were lysed for protein extraction. Fig. 4a: CD11b expression was measured by Western blotting analysis. Fig. 4b: The ratio of densitometry values of CD11b and *β*-actin was normalized to each respective control group. Results were the mean ± S.D. from three independent experiments performed in triplicate. *P<0.05 compared with the TET(−)LPS(+) group.

### 3.3 TET attenuated the production of IL1β and TNFα in BV2 cells

Cells were pretreated with different concentrations of TET for 2 hours (0.1 µM, 0.5 µM and 1 µM), and stimulated by LPS (1 µg/ml) for an additional 24 hours. Finally, the cells were lysed for the extraction of total RNA. The mRNA expression levels of IL1*β* and TNFα were measured by real-time RT-PCR.

As shown in Fig. 5a–5b, LPS stimulation remarkably increased the mRNA expression of IL1*β* and TNFα. However, TET pretreatment markedly suppressed these effects. Moreover, consistent with the changes in mRNA, the productions of mature IL1*β* and TNFα were significantly up-regulated after 24 hours of LPS stimulation, but was inhibited by TET pretreatment(Fig. 5c–5d).

**Figure 5:** The expression of IL1β and TNFα was attenuated by TET in BV2 cells. BV2 cells were treated with TET at working concentrations for 2 h. Then, LPS was added to each plate and incubated at 37°C for an additional 24 h. Then, the supernatant was collected and stored at −80°C for further ELISA assay. The cells were lysed for RNA extraction. Fig. 5a–5b: The mRNA expression of IL1β and TNFα was determined by real-time RT-PCR. Fig. 5c–5d: The production of IL1β and TNFα was measured by enzyme-linked immunosorbent assay (ELISA). Results were the mean ± S.D. from three independent experiments performed in triplicate. * *P*<0.05 compared with the LPS group.

### 3.4 TET suppressed LPS-induced microglia activation through the NF-κB and ERK signaling pathways

The NF-κB pathway and MAPK pathway have been shown to play vital roles in LPS-induced cytokine expression [30]. In this study, we investigated the influence of TET on NF-κB and MAPK activity in BV2 cells.

#### 3.4.1 Role of NF-κB in the effect of TET on LPS-induced microglia activation

Phospho-p65 and phospho-IKK were considered to be indicators of NF-κB activation. As shown in Fig. 6, the expression levels of phospho-p65 and phospho-IKK were significantly increased in the LPS group, whereas TET pretreatment remarkably suppressed these effects in a dose-dependent manner.

**Figure 6:** Effect of TET on LPS-stimulated NF-κB activity in BV2 cells. BV2 cells were treated with TET at working concentrations for 2 h. Then, LPS was added to each plate and incubated at 37°C for an additional 24 h. Then, the cells were lysed for protein extraction. Fig. 6a: p-p65, p65, p-IKK, IKK, and *β*-actin expression were measured by Western blotting analysis. Fig. 6b–6c: The ratio of densitometry values of total and phosphorylated protein was normalized to each respective control group. *β*-actin was applied as the internal control. Results were the mean ± S.D. from three independent experiments performed in triplicate. * *P*<0.05 compared with the LPS group.

#### 3.4.2 Role of the ERK pathway in the effect of TET on LPS-induced microglial activation

Next, we examined MAPK activity in BV2 cells. MAPKs comprise three major signaling molecules: extracellular signal-regulated kinase 1/2 (ERK 1/2), p38 MAPK, and c-Jun N-terminal protein kinase (JNK). Activation of MAPKs was measured by Western blot using phospho- or the total form of antibodies against ERK 1/2, p38 MAPK, and JNK. As shown in Fig. 7, phospho-ERK 1/2 was significantly increased in the LPS group. TET significantly inhibited these effects in a dose-dependent manner, while the phosphorylation of JNK and p38 were not influenced. We also noticed that the levels of the total forms of ERK 1/2, JNK, and p38 were not affected.

**Figure 7:** Effect of TET on LPS-stimulated MAPK activity in BV2 cells. BV2 cells were treated with TET at working concentrations for 2 h.Then, LPS was added to each plate and incubated at 37°C for an additional 24 h. Thereafter, the cells were lysed for protein extraction. Fig. 7a: Western blot assay was performed to evaluate the expression of total and phosphorylated forms of ERK1/2, JNK, and p38. *β*-actin was applied as the internal control. Fig. 7b: The ratio of densitometry values of total and phosphorylated forms of the protein was normalized to each respective control group. *β*-actin was applied as the internal control. Results were the mean ± S.D. from three independent experiments performed in triplicate. * *P*<0.05 compared with the LPS group.

#### 3.4.3 The inhibitory effect of TET on activated microglia was abolished by ERK1/2 and NF-kB inhibitors

To clarify whether the inhibitory effect of TET on activated microglia is indeed mediated by ERK1/2 and NF-κB signal pathways, BV2 cells were pretreated with PD98059 (a MEK1/2 inhibitor, 10 µM, Beyotime, Haimen, China), BAY 11–7082 (an NF-κB inhibitor, 5 µM, Beyotime, Haimen, China) and different concentrations of TET for 2 hours, then stimulated with LPS for an additional24 hours. Thereafter, the cells were lysed for total RNA extraction. The mRNA expression levels of IL1β and TNFα were monitored by real-time RT-PCR.

As shown in Fig. 8, the mRNA expression levels of IL1*β* and TNFα were remarkably increased in the LPS group.PD98059 and BAY 11–7082 dramatically inhibited this effect, and TET failed to show any additive effect.

**Figure 8:** Effect of PD98059 and BAY 11–7082 on IL1β and TNFα expression in LPS-induced microglial activation. In order to clarify whether the inhibitory effect of TET on activated microglia is really mediated by ERK1/2 and NF-κB signaling pathways, BV2 cells were pretreated with PD98059, BAY 11–7082, and working concentrations of TET for 2 hours, then stimulated with LPS for an additional 24 hours. Then, the cells were lysed to extract total RNA. The mRNA levels of IL1β (Fig. 8a) and TNFα (Fig. 8b) were measured by real-time RT-PCR. Results were the mean ± S.D. from three independent experiments performed in triplicate. * P<0.05 compared with the LPS+PD+BAY group.

## Discussion

Glaucoma is the second leading cause of irreversible visual impairment in the world [12]. Recent molecular analysis revealed that overactivated microglia were associated with the early stages of glaucoma. Microglia become activated prior to the evidence of the structural decline of RGCs [31]. Spatially, activated microglia were first localized to the optic nerve head and lamina around unmyelinated optic axons [31], [32], the presumed sites of initiation of optic neuropathy in humans [33], [34]. The pharmacologic regulation of microglial activity is a rational approach to the treatment of glaucoma. In the current study, we demonstrated that TET could inhibit microglial activation and attenuate the production of IL1β and TNFα through the NF-κB and ERK 1/2 signaling pathways. Moreover, our previous studies suggested that TET has beneficial effects in lowering intraocular pressure in a rat glaucoma model [35], and TET also could protect RGCs from ischemic injury in vitro and in vivo [36]. Thus, TET might be a promising candidate for glaucomatous therapy.

Because of the low cell number and time-consuming techniques that are required to cultivate primary microglia cultures, an immortalized BV2 microglia cell line has been utilized extensively in research related to neurodegenerative disorders. They have similar activation markers, motility, releasable factors and phagocytic function as those of primary microglia. CD11b is a molecular marker used in microglia identification. Previous studies suggested that CD11b took part in the pathologic process of animal models of glaucoma, deleting the CD11b gene prevented microglial activation and blocked pathophysiological effects [37]. Moreover, Zhang et al. [29] reported that the microglial activation induced by LPS are always accompanied by the up-regulation of CD11b. In this study, we found that LPS stimulation remarkably increased CD11b expression, but TET pretreatment abolished this effect in a dose-dependent manner. Additionally, we found that (94.5±2.6)% of BV2 cells displayed round or amoeboid shapes in the LPS group, but fewer in the 0.5 µM and 1 µM TET group (*P* = 0.045, *P* = 0.033, respectively). Therefore, we recognized that LPS-induced microglial activation was partially blocked by TET. However, morphological change has low sensitivity and specificity in evaluating the different functions of activated microglia in vitro. Chhor et al. [38] suggested that microglia exhibited four activated phenotypes: classically activated M1 with cytotoxic properties; M2a with an alternate activation and involvement in repair and regeneration; M2b with an immunoregulatory phenotype, and M2c with an acquired deactivating phenotype. They are characterized by a battery of phenotype markers and protocols for evaluating the functional outcome for screening novel neuroprotectants. This study gave us a comprehensive concept of the different phenotypes of microglial activation, and the effect of various doses of TET on LPS-induced M1 phenotype needs to be further investigated.

Activated microglia produce numerous pro-inflammatory cytokines, which are thought to contribute to the progression of glaucoma [37], [39], [40], [41], [42], [43]. Among these cytokines, IL1β has been suggested to play a central role in the immune response of glaucoma patients [39], [44]. Zhang et al. [45] reported that the over expression of IL1β could lead to optic nerve damage by increasing the synthesis of matrix mellanoproteinase-9 in mouse model of glaucoma, intravitreal injection of IL1 receptor antagonist could attenuate this effect. IL1β has also been reported to increase the generation of reactive oxygen species [35] and nitric oxide synthesis [46], [47] and is implicated in RGC damage leading to neurodegeneration. TNFα is another prominent pro-inflammatory mediator. Previous studies reported that the up-regulation of TNFα and its receptor were involved in the neurodegenerative process of glaucoma [48], [49]. Further in vitro studies also demonstrated that anti-TNFα could attenuate the RGC apoptosis induced by ischemia or elevated hydrostatic pressure [50]. Therefore, IL1β and TNFα are novel therapeutic targets for the treatment of glaucomatous optic neuropathy. Xue et al. [23] first reported that TET could suppress the production of TNFα and IL6 in LPS-induced microglial activation. They isolated rat primary microglia and pretreated them with TET in relatively high concentrations (25 µmol/Land 50 µmol/L) for 2 hours, after which they were stimulated using LPS (1 µg/ml). They found that TET pretreatment significantly inhibited the LPS-induced microglial activation. Interestingly, in our study, we found that TET with a concentration beyond 2 µmol/L might lead to cell apoptosis and affect cell viability. This paradox may be attributed to the different suppliers of TET or different cell types used in each experiment. Another study also reported similar results: in a fibrillar amyloid-β (fAβ)-induced microglial activation model, TET with different concentrations (0.1 µmol/L to 5 µmol/L) decreased the production of TNFα and IL1β in a dose-dependent manner. This study also found that TET did not influence the phagocytosis of microglia [22]. Consistent with previous studies, we found that TET significantly suppressed the expression of IL1*β* and TNFα both at the transcription and translation levels. Furthermore, the CCK-8 assay indicated that TET at optimal concentrations (0.1 µmol/L to 1 µmol/L) did not affect cell viability. Thus, the inhibitory effects of TET were not due to cytotoxicity. Therefore, we suggested that TET could attenuate the production of IL1β and TNFα in BV2 cells.

NF-κB is a key transcription factor that has been shown to regulate the expression of pro-inflammatory mediators and enzymes involved in the neurodegenerative process of glaucoma [51], [52], [53]. It is typically a heterodimer composed of p65 and p50 subunits. Inactive NF-κB complexes are located in the cytoplasm by binding to IκB (inhibitor of NF-kB) [54]. Once activated, IκB is quickly phosphorylated and degraded, allowing NF-κB to translocate to the nucleus, where it can bind to specific DNA sequences located in the promoter regions of target genes and activate gene transcription. Phosphorylation of IKK is a restriction step of NF-κB activation, and initiates the phosphorylation and degradation of IκB [43]. Thus, inhibiting the NF-κB signaling pathway may have beneficial effects. Xue et al. [23] found that TET dramatically abolished NF-κB-specific binding and suppressed the production of inflammatory mediators in rat primary microglial cells. He concluded that TET suppressed the production of inflammatory mediators by blocking the NF-κB signaling pathway. He et al. [22] reported that TET remarkably reduced the expression of phospho-p65 and proinflammatory cytokines in activated BV2 microglia. TET also has been proven to intervene with NF-κB activation and nuclear translocation in human peripheral blood T cells [55]. In our study, we found that the NF-κB signaling pathway was significantly activated after LPS stimulation, whereas TET pretreatment remarkably suppressed the phospho-p65 and phospho-IKK expression in BV2 cells. Our findings indicate that inhibition of the NF-κB signaling pathway maybe one of the mechanisms responsible for the reduction of proinflammatory cytokines.

In addition, the MAPK signaling pathway has been reported to play a pivotal role in the regulation of COX-2, NO, PGE2 and pro-inflammatory cytokine expression by controlling the activation of NF-κB in activated microglia [56], [57]. Jeonget al. [58] showed that the anti-inflammatory effect of α-galactosylceramide was mediated by the inhibition of p38 MAPK activation in activated BV2 cells. Kim et al. [25] showed that floridoside inhibited p38 and ERK 1/2 phosphorylation but not JNK in LPS-stimulated BV2 cells, while Dong et al. [59] showed that oxymatrine significantly inhibited all of the MAPKs, including ERK, p38, and JNK in LPS-induced BV2 cells. Up to now, no one has reported whether TET can affect the MAPK signaling pathway in activated microglia. Our study revealed that the phospho-ERK 1/2 was markedly suppressed by TET in a dose-dependent manner, while the phosphorylation of JNK and p38 were not influenced. This is the first study to report that TET can inhibit the MAPK signaling pathway in LPS-induced microglial activation. Additionally, PD98059 (an ERK1/2 inhibitor) and BAY 11–7082 (a NF-κB inhibitor) dramatically suppressed LPS-induced mRNA expression (IL1*β* and TNFα), and TET failed to show any additive effect. This result indicates that ERK 1/2 and NF-κB activation mainly regulates IL1β and TNFα induction in LPS-stimulated microglial cells and that TET typically exerts their inhibitory effects by inhibiting ERK 1/2 and NF-κB phosphorylation.

In conclusion, our results show that TET can effectively suppress microglial activation and inhibit the expression of IL1*β* and TNFα by regulating NF-kB and ERK signaling pathways. Together with our previous studies, we suggest that TET would be a promising candidate to effectively suppress overactivated microglia and alleviate neurodegeneration in glaucoma. Further in vivo studies are necessary to evaluate the response of activated microglia and the interaction between neurons and microglia due to TET pretreatment.
